# The therapeutic landscape for COVID-19 and post-COVID-19 medications from genetic profiling of the Vietnamese population and a predictive model of drug-drug interaction for comorbid COVID-19 patients

**DOI:** 10.1016/j.heliyon.2024.e27043

**Published:** 2024-03-05

**Authors:** Thien Khac Nguyen, Giang Minh Vu, Vinh Chi Duong, Thang Luong Pham, Nguyen Thanh Nguyen, Trang Thi Ha Tran, Mai Hoang Tran, Duong Thuy Nguyen, Nam S. Vo, Huong Thanh Phung, Tham Hong Hoang

**Affiliations:** a Center for Biomedical Informatics, Vingroup Big Data Institute, Hanoi, Viet Nam; b GeneStory JSC, Hanoi, Viet Nam; c Faculty of Biotechnology, Hanoi University of Pharmacy, Hanoi, Viet Nam

**Keywords:** COVID-19 drugs, Post-COVID-19 drugs, Pharmacogenomics, Drug interactions, Chronic diseases, Vietnamese population

## Abstract

Despite the raised awareness of the role of pharmacogenomic (PGx) in personalized medicines for COVID-19, data for COVID-19 drugs is extremely scarce and not even a publication on this topic for post-COVID-19 medications to date. In the current study, we investigated the genetic variations associated with COVID-19 and post-COVID-19 therapies by using whole genome sequencing data of the 1000 Vietnamese Genomes Project (1KVG) in comparison with other populations retrieved from the 1000 Genomes Project Phase 3 (1KGP3) and the Genome Aggregation Database (gnomAD). Moreover, we also evaluated the risk of drug interactions in comorbid COVID-19 and post-COVID-19 patients based on pharmacogenomic profiles of drugs using a computational approach. For COVID-19 therapies, variants related to the response of two causal treatment agents (tolicizumab and ritonavir) and antithrombotic drugs are common in the Vietnamese cohort. Regarding post-COVID-19, drugs for mental manipulations possess the highest number of clinical annotated variants carried by Vietnamese individuals. Among the superpopulations, East Asian populations shared the most similar genetic structure with the Vietnamese population, whereas the African population showed the most difference. Comorbid patients are at an increased drug-drug interaction (DDI) risk when suffering from COVID-19 and after recovering as well due to a large number of potential DDIs which have been identified. Our results presented the population-specific understanding of the pharmacogenomic aspect of COVID-19 and post-COVID-19 therapy to optimize therapeutic outcomes and promote personalized medicine strategy. We also partly clarified the higher risk in COVID-19 patients with underlying conditions by assessing the potential drug interactions.

## 1 Introduction

The Coronavirus disease 2019 (COVID-19) pandemic caused by the severe acute respiratory syndrome coronavirus 2 (SARS-CoV-2) has been posing a major challenge to global healthcare systems with various detrimental impacts on public health and clinical practice in many countries and territories including Vietnam [1,2]. To date, there have been many types of available repurposed and novel drugs for COVID-19 treatment [[3], [4], [5]]. There has been several drugs that was approved for used in COVID-19 patients, including antiviral agents remdesivir, nirmatrelvir combined with ritonavir, and two immune modulators baricitinib and tocilizumab [3]; however, their adverse effects should not be ignored. ADRs attributed to COVID-19 drugs might be one of the leading causes of morbidity and mortality in COVID-19 patients, especially elderly individuals and those with comorbidities [6,7]. Due to polypharmacy and age-related degradation of organ functions, such patients could be highly susceptible to drug-drug interactions (DDIs) and serious toxicities of COVID-19 therapies, leading to a significantly higher mortality rate in some populations [8,9].

Moreover, most patients with COVID-19 recover after acute infection with SARS-CoV-2, but a proportion report ongoing health problems. One study found that up to 70% of individuals at low risk of mortality from COVID-19 have impairment in one or more organs (i.e., heart, lungs, kidneys, liver, pancreas, or spleen) four months after initial COVID-19 symptoms [10]. Four common conditions reported are chronic fatigue syndrome, manipulations in the respiratory system, manipulations in the cardiovascular system, and mental symptoms [11]. The multiple drugs used for managing these various conditions also pose a danger of ADRs and DDIs.

Pharmacogenomics (PGx) is the discipline of science that could clarify the impacts of genetic polymorphisms on the inter-individual variability of drug response. Genetic factors have been reported to modulate the pharmacokinetic (PK) and pharmacodynamic (PD) properties of drugs and consequently, they are partly responsible for the unpredictable therapeutic outcomes and ADRs [12,13]. The understanding of variants located on genes encoding the elements participating in PK/PD pathways of COVID-19 and post-COVID-19 drugs (such as enzymes, transporters, targets, and carriers) enables clinicians to choose proper treatment regimens for individuals in order to improve the therapeutic outcomes and minimize ADRs [14]. In addition to assistance in drug choosing, the understanding of genes and proteins involved in PK and PD of drugs and their polymorphic variants in patients could help to predict risks of DDIs in those with polypharmacy such as COVID-19 or post-COVID-19 patients. However, gene variations affecting the response of patients to COVID-19 pharmacotherapies have not been clinically studied, so pharmacogenomic data for these drugs is extremely scarce [12]. In spite of the raised awareness of the role of PGx in personalized medicines for COVID-19 [15,16], only one study on the actionable genetic variants relating to COVID-19 drugs has been done on the Indian population [17]. There has not been any publication on the PGx data relating to post-COVID-19 medications to date.

Data from whole genome sequencing of human populations across the world has greatly contributed to the attempts to promote personalized medicine and provide population-specific evidence to help clinicians in practice [18]. In 2021, Vingroup Big Data Institute (VinBigdata) officially announced the completion of the 1000 Vietnamese Genomes Project (1KVG) with a scale of 1008 genomes of healthy individuals sequenced [MASH portal. https://genome.vinbigdata.org/]. 1KVG is the first genome-wide dataset ensuring the representativeness and universality of the Vietnamese population, consistent with the geographical population and gender distribution. Exploiting information on PGx variants from this database can offer better understanding and clinical practice in the management of COVID-19.

This study focused on understanding Vietnamese genetic variations and alleles that are associated with the safety and effectiveness of drugs administered during and post-COVID-19 management. Besides, we also provide a holistic panorama of potential DDIs among COVID-19 therapies and drugs used in the treatment of comorbidities to inform clinicians to make more accurate decisions and potentially improve therapeutic outcomes.

## 2 Materials and methods

### 2.1 Study population and datasets

The 1000 Vietnamese Genomes Project (1KVG): Participants of the 1KVG project were recruited from Kinh ethics all over Vietnam, from the North to the South, and equally divided among both sexes. The genetic variants and their allele frequencies (AFs) in the Vietnamese population were collected from the Variant Calling Format (VCF) of 1008 whole genome sequences of unrelated healthy Vietnamese individuals. All participants in the project provided written informed consent. The study complied with the Declaration of Helsinki and was approved by the Ethics Committee of the Vinmec International Hospital (543/2019/QƉ-VMEC). The variant file included genotype information for 49,201,339 variants [MASH portal. https://genome.vinbigdata.org/]. The variants are annotated according to the *GRCh38* human reference genome.

The WGS data of 2504 unrelated individuals of different populations in the world in the 1000 Genomes Project Phase 3 (1KGP3) [19] and the Genome Aggregation Database (gnomAD) [20] containing 76,156 genomes of diverse ancestries were used for the comparison with the 1KVG.

### 2.2 Medication of choice

Information on the medications to manage COVID-19 was obtained from the guidelines issued by WHO [5,21], the US National Institute of Health [3], along with the 8th guidelines for the diagnosis and treatment of COVID-19 released by the Vietnam Ministry of Health [4]. Information on the medications used for post-COVID-19 conditions was collected from the guidelines issued by WHO [21], the U.K National Institute for Health and Care Excellence (NICE) [22], along with the guidelines for the diagnosis and treatment of post-COVID-19 for adults [11] and children at home [23] released by the Vietnam Ministry of Health.

### 2.3 Construction of the comprehensive landscape of COVID-19 drugs-related pharmacogenomic variants from PharmGKB and DrugBank in the Vietnamese population

The whole process of the construction of COVID-19 drug-related pharmacogenomic variations for the Vietnamese population was displayed in Fig. 1. PharmGKB clinical annotations [24,25] of all levels including SNP/indels, star alleles, and HLA alleles related to COVID-19 and post-COVID-19 drugs in our list were curated. Then, we identified the number of variants carried by Vietnamese people in the 1KVG for every single drug to show the comprehensive pharmacogenomic landscape of COVID-19 and post-COVID-19 drugs in the Vietnamese population. These results were presented by median and the range of the number of variants carried by 1008 participants in the 1KVG and were also depicted by a violin plot with a boxplot inside. The Stargazer [26] was used to call the star alleles of PGx genes from the whole genome variation data (VCF file) of the 1KVG and 1KGP3 databases. xHLA [27] was the bioinformatics tool used for the HLA typing which could generate four-digit resolution for both class I and II HLA genes.

**Fig. 1:** Diagram presenting the process of the construction COVID-19 drugs-related pharmacogenomic variations for the Vietnamese population. 1KVG: 1000 Vietnamese Genomes Project, AF: Allele frequency, SNP: single nucleotide polymorphism.

Information on drug cellular transporters, metabolic enzymes, targets, and carrier proteins within the blood and biological fluids of COVID-19 and post-COVID-19 medications were retrieved from the DrugBank [28]. All variants located in the genes encoding these elements were queried from the 1KVG database, then annotated by ANNOVAR using dbSNP v147 and RefGene annotations, and functional impacts of these variations were estimated using the SIFT [29], PolyPhen-2 [30], and MutationTaster [31,32]. The nonsynonymous exonic variants were predicted to be deleterious by at least two of the three tools including SIFT (Damaging), Polyphen2 (Damaging or Probably damaging), or Mutation Taster2 (Disease_causing).

The clinically deleterious variations predicted by two of the aforementioned sources with AF>1% in the 1KVG database were retained to establish a list of variants that have evidence to be associated with COVID-19 pharmacotherapies.

### 2.4 Statistical analysis

To reveal the distinction in genetic risks related to COVID-19 and post-COVID-19 drugs between the Vietnamese population and other populations, we performed a Fst analysis for the entire identified pharmacogenomic variants list using the PLINK v1.09. The higher Fst, the greater distinction between populations. The weighted Fst scores for each population pair were plotted using a heatmap.

We also used Fisher's exact test to assess the significant differences between the Vietnamese and other super cohorts from the global populations (derived from both the 1KGP3 and the gnomAD) in allele frequencies of genetic variations (PharmGKB level 1A/B and 2A/B) which are relevant to COVID-19 and post-COVID-19 therapies. The p-value <0.05 in the Fisher exact test showed a significant difference in AF between the two populations.

### 2.5 Drug-drug interaction analysis

We performed interaction analyses to identify potential DDIs among the COVID-19 treatment medications, as well as between the COVID-19 drugs and the drugs commonly used in the treatment of the three chronic diseases (cardiovascular diseases, diabetes, and cancers) to explore the reason underlying the high risk of suffering from DDI in COVID-19 patients. The computational prediction of DDIs based on the drug functional similarity method which was previously described by Ferdousi et al. [33]. Five types of binary vectors including carrier, transporter, metabolic enzyme, target (CTET) vectors as well as a comprehensive vector consisting of all CTET elements were used for the analyses.

The information on drug-CTET element pairs was extracted from the DrugBank. The duplicated elements (if any) were removed from the list. Then, for each COVID-19-relating drug, 5 binary vectors were constructed. The length of vectors which was calculated from the total number of all pharmacogenes related to all investigated drugs expresses the total number of CTET elements participating in the pharmacodynamic (PD) and pharmacokinetic (PK) pathways of these drugs. For each drug, the value of each index of the vector was set at 1 if this element was involved in the drug's pathway, otherwise it was set at 0.

After the vector construction, drugs with zero vectors were eliminated. Then the similarity-measuring for all drug pairs was calculated using the Russell-Rao approach, which was reported to be the best similarity-measuring tool for analyzing the probability of DDIs [33]. The Russell-Rao similarity-measuring was calculated by the equation:

$$S=\frac{x^{t}y}{d}$$

In which: x and y are binary feature vectors of length d. The vector multiplication of x and y x^t^y indicates the positive matches which were equivalent to the number of biological elements shared among every two drugs). A drug pair will be identified as a potential DDI if its similarity value is > 0. The construction and similarity measurement of vectors are summarized in Fig. 2.

**Fig. 2:** **Vectors construction for each drug pair.***Red circles show the shared element between drug pair (CTET: carrier, target, enzyme and transporter). The upper panel depicts the comparison of each element (i.e. carrier, target, enzyme and transporter) between two given drugs and the lower depicts the comparision of hybrid vectors including all elements between two given drugs.*

The higher similarity values, the greater the possibilities of interactions. However, it should be noted that the level of similarity does not directly refer to the level of detrimental impacts.

The potential interactions between two COVID-19 drugs through enzymes, targets, transporter, and carrier were illustrated by a network displaying the shared components in these drugs' pathways.

### 2.6 Data visualizations

All the data visualized plots were generated by the R 3.6.3 and RStudio April 1, 1717. Cytoscape is used to display the drug-gene interactions in the network. Sizes of the gene labels are proportional to the degree of the node (number of drugs sharing this gene in their pathway), whereas the drug labels are sized according to the number of pharmacogenes in its pathways.

## 3 Results

### 3.1 Pharmacogenomics of COVID-19 medications in Vietnamese people

According to the guidelines for the COVID-19 treatment [[3], [4], [5]], there are 50 drugs currently involved in COVID-19 therapy (Table S1). These drugs could be classified into four categories: Cause treatments (antiviral agents/antiviral antibodies/interleukin inhibitors), corticoids, antithrombotic agents, and treatments for superinfection. 19 out of 50 drugs have at least one PharmGKB clinical annotation, whereas 37 drugs are associated with pharmacogenes listed by the DrugBank database. Totally, 9 out of 50 drugs do not have any pharmacogenomic information available.

### 3.2 Actionable pharmacogenomic variations relating to the COVID-19 medication in Vietnamese people

We obtained a total of 181 clinical annotations for all levels from PharmGKB that are related to our COVID-19 drug list. They consisted of 117 single nucleotide polymorphisms (SNPs) of which 2 SNPs located in mtDNA were excluded due to the unavailability in the population genetic databases. Besides, our list also included 23 star-alleles of the Cytochrome P450 (CYP) superfamily, the *NAT2* gene, and 11 *HLA* alleles have been reported to be associated with differential responses to drugs used for COVID-19 treatment at different levels (Table S2).

The genetic impacts on different drug groups were very distinct, which could be seen due to the difference in the number of clinically annotated variants carried by the Vietnamese population (Fig. 3). Among the drugs used in COVID-19 treatment, the pharmacogenomic profile of antithrombotics was most thoroughly studied [12]. Warfarin was reported to be associated with the largest number of variants (89 variants for 4 levels), while new oral anticoagulants (NOAC) (apixaban, rivaroxaban, and dabigatran) also have numerous variants associated with their efficacy and/or toxicity [24]. In the current study, all Vietnamese people carry more than one deleterious variant relating to the anticoagulant agents (Warfarin: 25.5 (range, 14–34), Rivaroxaban: 1 (range, 0–2) Apixaban: 1.5 (range, 0–3), Dabigatran: 2 (range, 0–4)).

**Fig. 3:** **Violin plot displaying the number of actionable pharmacogenetic variations relating the COVID-19 medications in the 1KVG**. *Inside boxplot present the Median, Quartiles and Interquartile Range to describe the distribution of number of clinical annotated variants carried by Vietnamese people.*

Regarding the causal treatment medications, only two agents (ritonavir and tocilizumab) had clinical annotations in PharmGKB. Variants affecting the efficacy and/or toxicity of both drugs are quite common in the Vietnamese population with the median of the related SNP number carried by Vietnamese people being 3 (range, 0–7) for tocilizumab and 9.5 (range, 4–15) for ritonavir.

Two corticosteroid agents have been used in the management of COVID-19 in Vietnam with very different PGx profiles. Dexamethasone has been widely used in severe COVID-19 patients, but the median of deleterious variants carried in the Vietnamese population is 3.5 (range, 0–7) whereas there was only one variant reported to be related to methylprednisolone, notably the variant was carried by 86.2% of the population.

There is much less evidence regarding variants that have been reported to be related to the response of antibiotics used for superinfection treatment, especially the beta-lactams, such as ceftriaxone, cefotaxime, amoxicillin/clavulanic acid …. However, most Vietnamese people carry at least one risk variant related to co-trimoxazole (95.2%) and voriconazole (95.2%).

### 3.3 The identification of novel variants that potentially influence the response to COVID-19 drugs

In addition to the variants that were annotated by PharmGKB, we identified 26 more variants in the Vietnamese population that were predicted by the SIFT, Polyphen-2, and Mutation Taster to affect the efficacy/toxicity of COVID-19 drugs (Table S3).

Regarding metabolic enzymes, we identified a variant (rs3826190) with an allele frequency of 3.2% in the Vietnamese population. The variant was located in the *CES1* gene coding a hydrolyzing enzyme that is responsible for the activation of remdesivir [34]. Besides, there are 2 missense variants in the *CYP2A6* gene including the rs28399468 which was comprised of the CYP2A6*8 allele and the rs5031016 which was comprised of the CYP2A6*7 allele. These two variants with allele frequency in the 1KVG of 4.5% and 13.0%, respectively might partly influence the metabolism of two corticoids including methylprednisolone and dexamethasone.

In terms of transporters, we detected that the rs11568658 variant of the *ABCC4* gene which accounts for 10.6% of the 1KVG, might have impacts on the function of the multidrug resistance-associated protein MRP4, thereby affecting the therapeutic response of remdesivir [35,36]. We also found a common SNP in the *SLC15A2* gene (rs1143671) which accounts for 63.3% of the Vietnamese population along with another variant in the *SLC15A1* gene (rs2274827) with AF of 10.5%. These two variants could disrupt the transportation of many beta-lactam antibiotics such as ampicillin, cefepime, cefotaxime, and ceftriaxone [37].

### 3.4 The similarity and distinction in pharmacogenomics relating to COVID-19 drugs between the Vietnamese population and other populations

There is an obvious difference between populations in pharmacogenomic structure related to COVID-19 drug response over the world (Fig. 4). As expected, the Vietnamese cohort show the highest similarity in genetic structure with the East Asian populations with the Fst of 0.037 when compared with the Japanese population (JPT) and 0.029, 0.035, and 0.030 when compared with the Chinese populations of CDX, CHB, and CHS, respectively. Meanwhile, African is the population that showed the most distinct in pharmacogenomics related to COVID-19 drugs in comparison with the Vietnamese population (Fst of 0.182, 0.181, 0.191, 0.184, 0.188, 0.194, and 0.180 when compared with the ACB, GWD, ESN, MSL, YRI, LWK, and ASW populations).

**Fig. 4:** **Heatmap displaying Fst scores for 1KVG versus 1KGP3 populations using COVID-19 drugs-related variants. 1KVG*: 1000 Vietnamese GenomesProject, East Asian****(CHS: Han Chinese South; CDX: Chinese Dai in Xishuangbanna, China; CHB: Han Chinese Beijing, China; JPT: Japanese in Tokyo, Japan),****South Asian****(PJL: Punjabi in Lahore, Pakistan; BEB: Bengali in Bangladesh; STU: Sri Lankan Tamil in the U.K.; ITU: Indian Telugu in the U.K.; GIH: Gujarati Indians in Houston, Texas, USA);****European****(GBR: British From England and Scotland; FIN: Finnish in Finland; IBS: Iberian Populations in Spain; CEU: Utah residents (CEPH) with Northern and Western European ancestry;TSI: Toscani in Italia),****American****(PUR: Puerto Rican in Puerto Rico; CLM: Colombian in Medellín, Colombia; PEL: Peruvian in Lima Peru; MXL: Mexican Ancestry in Los Angeles CA USA),****African****(ACB: African Caribbean in Barbados; GWD: Gambian in Western Division - Mandinka; ESN: Esan in Nigeria; MSL: Mende in Sierra Leone; YRI: Yoruba in Ibadan, Nigeria; LWK: Luhya in Webuye, Kenya; ASW: African Ancestry in SW, USA.*

Regarding the variations at level 1 and 2 of the PharmGKB recommendations, AF of these genetic variations significantly varies between the Vietnamese cohort and other populations in the world (Fig. 5). There are various curated PharmGKB level 1 and level 2 annotations that were associated with warfarin and acenocoumarol, including the variations in the *CYP2C9*, *VKORC1*, and *CYP4F2* genes. Most Vietnamese people carry the normal-function allele CYP2C9*1 with a frequency of 97.1%, which is significantly higher than the global population (1KGP3_AF = 84.6%). Much more attention should be paid to the variants of the *VKORC1* gene encoding the Vitamin K epoxide reductase complex subunit 1 protein, the target of the vitamin K antagonist – VKA. Variants located in the *VKORC1* gene have been well-documented to affect the response of patients to the classic anticoagulants [38]. Among those, three variants including the rs8050894 (PharmaGKB level 1B), rs9923231 (level 1A), and rs9934438 (level 1B) are the most common variants in the Vietnam population with the prevalence of 85.1%, 85.0%, and 85.1%, respectively, which are approximately two-times higher than the prevalence in the general global population (41.6%, 35.6%, 35.6%, respectively). These variants could lead to a decreased expression of the VKORC1, resulting in a lower dosage requirement of warfarin [39]. In contrast, the AF of the rs2359612 (level 1B) and rs2884737 (level 2A) are significantly lower compared to the global populations (p < 0.001, Fisher's test). In particular, the prevalence of the rs2359612 is 14.9% in the Vietnamese people, whereas it is extremely high in the South Asian populations (AF = 85.5%) and the global population (AF = 61.0%). The presence of the T nucleotide at this locus also leads to a lowered gene expression which then subsequently is associated with a decrease in warfarin dose requirement [40]. The enzyme coded by the *CYP4F2* gene is responsible for the metabolism of vitamin K to hydroxy-vitamin K1 which can not enter the vitamin K cycle [41]. The rs2108622 variant on this gene is well-known to be associated with warfarin dosing (PharmGKB level 1A) [42]. The frequency of this variant was similar between the Vietnamese and the global population (1KVG = 0.202, 1KGP3_ALL = 0.237). A study by Caldwell et al. calculated that each T allele of the rs2108622 is associated with a 4–12% increase in warfarin dose, so that a patient with the TT genotype could require an approximate 1 mg/day higher dose of warfarin compared to a patient with the homogenous wildtype genotype [42].

**Fig. 5:** **Allele frequencies of variations associated with COVID-19 therapies (Level 1 & 2 in PharmGKB) and the comparisons between the 1KVG and other populations derived from 1KGP3 and gnomAD**. *Red dots depict non-significant difference in AF compared to* 1KVG *(Fisher's exact test p ≥ 0.05), blue dots depict significant difference in AF compared to* 1KVG *(p < 0.05). The dot size are proportional to the AF of variations. 1KGP3_ALL: 1000 Genomes Project Phase 3, gnomAD_ALL: The Genome Aggregation Database, AFR: African, AMR: American, ASJ: Ashkenazi Jewish, EAS: East Asian, EUR: European, FIN: Finnish, NFE: Non-Finnish European, SAS: South Asian, OTH: Other population.*

The *CYP2C19* gene encodes an enzyme significantly involved in the metabolism of voriconazole which is used for superinfection treatment. A majority of participants in the 1KVG carry the normal function allele CYP2C19*1 (AF = 64.3%) whereas the CYP2C19*17 allele with increased function phenotype account for only 1.1% of the Vietnamese population. 29.4% and 5.2% of the Vietnamese population carry the no-function alleles CYP2C19*2 and CYP2C19*3, respectively. Such AF was significantly higher than that of the global cohorts (22.1% and 1.4%, respectively in the 1KGP3_ALL). This fact raises a great concern for the Vietnamese people when using voriconazole for antifungal treatment. The deficiency of CYP2C19 activity results in a longer time of exposure to voriconazole and consequently, causes various adverse events such as hepatotoxicity or visual disturbances [43,44].

A total of 6 *HLA* alleles related to co-trimoxazole response have level 2A/B evidence. Among them, HLA-B*15:02 and HLA-C*08:01 were shown the highest rate in the population with a prevalence of 19.1% and 13.5%, respectively, which are significantly higher than those in the global population (1KGP3_ALL: 2.4% and 3.1%, respectively). Both have been demonstrated to be associated with the risk of Stevens-Johnsons syndrome or Toxic Epidermal Necrolysis (SJS/TEN) when using trimethoprim/sulfamethoxazole [45,46].

## 4 Pharmacogenomics of the post-COVID-19 medications in Vietnamese people

There are 83 agents which were used for post-COVID-19 management (Table S4). These drugs were administered for treating four common conditions after SARS-CoV-2 infection including chronic fatigue syndrome, manipulations in the respiratory system, manipulations in the cardiovascular system, and mental syndromes.

### 4.1 Actionable pharmacogenomic variations relating to the post-COVID-19 medications in Vietnamese people

A total of 881 clinical annotations of all levels from PharmGKB was associated with the post-COVID-19 therapy, of which, 331 SNPs, 93 star-alleles, and 4 *HLA* alleles were reported to be associated with differential response to drugs used for post-COVID-19 treatment (Table S5).

Among these agents, drugs for major depressive and anxiety disorders (e.g. duloxetine, risperidone, olanzapine, …) posed the highest risk for the Vietnamese population. For example, duloxetine – a serotonin and norepinephrine reuptake inhibitor (SNRIs) has a median number of related risk variants of 45.5 (range, 20–69). Aspirin which could be used in pain management and as an antiplatelet in several cardiovascular conditions also poses a remarkable genetic risk with a median of 30 (range, 18–44). Acetaminophen is the most popular OTC analgesic, especially for post-COVID-19 headache treatment, thanks to its safeness and effectiveness. However, the genetic profile of Vietnamese people may raise concerns about using acetaminophen with the median number of related risk variants carried by Vietnamese people being 7 (range, 3–11) (Fig. 6).

**Fig. 6:** **Violin plot displaying the number of actionable pharmacogenetic variations relating the post-COVID-19 medications in the 1KVG.***Inside boxplot present the Median, Quartiles and Interquartile Range to describe the distribution of number of clinical annotated variants carried by Vietnamese people.*

### 4.2 The identification of novel variants that potentially influence the response to post-COVID-19 drugs

Aside from the PharmGKB annotation, we reported a list of 73 potentially deleterious variants which were predicted to be associated with the response of post-COVID-19 medications (Table S6).

Relating to the targets of drugs used for cardiovascular disorders post-acute sequelae of SARS - CoV2 infection, a series of variants could alter the structure of the Calcium Voltage-Gated Channel Subunits, such as the rs181892888 (AF of 1.43%) and rs573493037 (AF of 1.33%) on the *CACNA1H* gene, the rs1799938 (AF of 11.62%) on the *CACNG1* gene, or the rs16023 (AF of 11.92%) on the *CACNA1A* gene, potentially affecting the efficacy/toxicity of the Calcium Channel Blockers. Amiodarone could be used in patients dealing with atrial or ventricular arrhythmia. The receptor encoded by the *PPARG* gene has been demonstrated to play an important role in amiodarone-induced pulmonary phospholipidosis [47]. We identified the rs11959820, a variant of the *PPARG* gene with a significant AF of 15.08% in the Vietnamese cohort, which could affect the structure of such receptor and thereby the toxicity of amiodarone. Moreover, a variant of the *HTR1D* gene (rs146071014 with AF of 1.7% in the Vietnamese population) could affect the structure of serotonine (5-HT) receptors, and probably be involved in extrapyramidal side effects of many antipsychotic medications [48].

In terms of transporters, the mentioned variants in *ABCC4* (rs11568658 with AF of 10.6%) could affect the response to many agents (NSAIDs, propranolol, verapamil, …) [49]. NSAIDs treatment could induce the overexpression of MRP4 encoded by *ABCC4* gene, resulting in platelet hyper-reactivity and eventually increasing cardiovascular risk [50]. Besides, the *SLC22A* family encodes the transporter hOCTs which are responsible for the transportation of an array of drugs [51,52]. Therefore, the observed variants on the *SLC22A1* gene (rs2282143 with AF of 10.8%) and the *SLC22A2* gene (rs316019 with AF of 85.3%) can disrupt the transportation of many drugs (such as flurazepam, antihistamines of the first generation, metoprolol, propranolol, …).

We also detected various variants on genes encoding enzymes involved in the metabolism of post-COVID-19 drugs. On the *CYP1A1* gene, we identified that the rs4646422 which comprised of the CYP1A1*13 allele with AF of 7.4%, and the rs180744198 with AF of 1.0% in the Vietnamese population could have effects on the biological activity of such metabolizer, resulting in the changes in bioavailability and eventually effectiveness of fluvoxamine, haloperidol, clozapine, melatonin, and amiodarone. The CYP2A6 participates in the metabolisms of many drugs that could be used in the post-acute sequelae phase of SARS-CoV-2 infection (e.g., vortioxetine, clozapine, amiodarone) [53]. The *CYP2A6* variants such as the rs5031016 which comprised the CYP2A6*7 allele with AF of 13.0% and rs28399468 which comprised of the CYP2A6*8, *10 alleles with AF 4.5% in the Vietnamese population were reported to be deleterious for the response of patients. Aside from the star-alleles of the Cytochrome P450 family which are responsible for phase 1 of drug metabolism, we also identify a number of variants located on the genes encoding phase 2 enzymes, such as *UGT1A1* (rs4148323 with AF of 10.5%), *UGT1A3* (rs45625338 with AF of 2.3%, rs45449995 with AF of 1.4%) and *UGT2B10* (rs1976666 with AF of 7.5%). Several angiotensin receptor blockers (ARBs) such as telmisartan are exclusively metabolized by the UGT enzyme family to become inactive metabolites [54]. Therefore, genetic mutations which increase or decrease the expression of these genes potentially impact the response of the related drugs. Moreover, these enzymes are potentially inhibited by various drugs (e.g., NSAIDs, losartan, telmisartan, etc), which may trigger adverse drug-drug interaction, leading to detrimental consequences. Additionally, we also identified a deleterious variant of the *CBR1* gene (rs117272030 found in 15.8% of the Vietnamese population) which potentially affects the metabolism of many xenobiotics, including haloperidol [55].

### 4.3 The similarity and distinction in pharmacogenomics relating to post-COVID-19 drugs between the Vietnamese population and other populations

Similar to COVID-19 drugs, there is also a significant difference in the genetic structure related to post-COVID-19 drug response (Fig. 7). However, compared to COVID-19, post-COVID-19 medications showed a lower inter-populations variability expressed by the lower Fst. The East Asian populations still have the most similar genetic profile to the Vietnamese people (Fst of 0.011, 0.016, 0.013, and 0.023 for the CDX, CHB, CHS, and JPT populations). The most distinct population is also African, but Fst index was lower than those of the COVID-19 medications (Fst of 0.141, 0.154, 0.150, 0.152, 0.155, 0.153, and 0.131 for the ACB, GWD, ESN, MSL, YRI, LWK, and ASW populations).

**Fig. 7:** **Heatmap displaying Fst scores for the 1KVG versus 1KGP3 populations using post-COVID-19 drugs-related variants. 1KVG*: 1000 Vietnamese Genomes Project, East Asian****(CHS: Han Chinese South; CDX: Chinese Dai in Xishuangbanna, China; CHB: Han Chinese Beijing, China; JPT: Japanese in Tokyo, Japan),****South Asian****(PJL: Punjabi in Lahore, Pakistan; BEB: Bengali in Bangladesh; STU: Sri Lankan Tamil in the U.K.; ITU: Indian Telugu in the U.K.; GIH: Gujarati Indians in Houston, Texas, USA);****European****(GBR: British From England and Scotland; FIN: Finnish in Finland; IBS: Iberian Populations in Spain; CEU: Utah residents (CEPH) with Northern and Western European ancestry;TSI: Toscani in Italia),****American****(PUR: Puerto Rican in Puerto Rico; CLM: Colombian in Medellín, Colombia; PEL: Peruvian in Lima Peru; MXL: Mexican Ancestry in Los Angeles CA USA),****African****(ACB: African Caribbean in Barbados; GWD: Gambian in Western Division - Mandinka; ESN: Esan in Nigeria; MSL: Mende in Sierra Leone; YRI: Yoruba in Ibadan, Nigeria; LWK: Luhya in Webuye, Kenya; ASW: African Ancestry in SW, USA.*

Regarding the variant at level 1 and level 2 of the PharmGKB recommendations, there is a significant distinction in the AF of identified variations between the 1KVG and other populations, which were mostly found with the CYP genes (Fig. 8). CYP2D6 polymorphisms are those with high-level evidence to affect the pharmacokinetic properties and toxicity of several drugs such as amitriptyline, codeine, serotonin selective reuptake inhibitors-SSRIs, and serotonin norepinephrine reuptake inhibitors-SNRIs, …) [[56], [57], [58]]. We found a significantly lower prevalence of the normal-function allele CYP2D6*1 in the Vietnamese cohort (2.6%), while its AF in the global population is about 42.7%. On the contrary, the severely decreased-function allele CYP2D6*10 is approximately 4.5-fold higher in the 1KVG (64.2%) than the 1KGP3_ALL (14.5%).

**Fig. 8:** **Allele frequencies of variations associated with post COVID-19 therapies (Level 1 & 2 in PharmGKB) and the comparisons between the 1KVG and other populations derived from 1KGP3**. *Red dots depict non-significant difference in AF compared to* 1KVG *(Fisher's exact test p ≥ 0.05), blue dots depict significant difference in AF compared to* 1KVG *(p < 0.05). The dot size are proportional to the AF of variations. 1KGP3_ALL: 1000 Genomes Project Phase 3, AFR: African, AMR: American, EAS: East Asian, EUR: European, SAS: South Asian.*

CYP2C19 is the major enzyme catalyzing the metabolism of the SSRIs and TCAs [58]. As described above, the Vietnamese population was at a higher risk related to *CYP2C19* metabolism because approximately one-third of the cohort carry the no-function allele (CYP2C19*2 and *3).

Regarding the HLA alleles, only HLA-DPB1*03:01 associated with toxicity of aspirin was classified in level 2B by PharmGKB [59]. The prevalence of this allele in the Vietnamese population is 5.2%, which is quite similar to other populations, such as East Asian, South Asian, and European cohorts with prevalence of 4.5%, 5.7%, and 5.1%, respectively.

## 5 Analysis of drug-drug interaction

### 5.1 DDIs relating to the COVID-19 medications

The two well-known genes, *CYP3C4* and *ABCB1* are the most shared pharmacogenes among the COVID-19 drugs [60,61]. Besides, other cytochrome P450 enzymes, such as CYP2C9, CYP2C19, and CYP3A5 also participate in PK/PD pathways of many drugs including ritonavir, fluconazole, apixaban, and rivaroxaban (Fig. 9). Based on the pharmacogene profile, by using a computational approach we detected 398 potential DDIs within the current COVID-19 drugs list (Table 1), suggesting a high probability of encountering DDIs in COVID-19 patients.

**Fig. 9:** **The network representation of the drug–gene interactions involved in COVID-19 therapy.***The drug and gene labels are colored in pink and green, respectively. The label sizes are proportional to the degree of this gene/drug.*

**Table 1:** Number of potential DDI pairs.

Underlying conditions	non-COVID-19	COVID-19	Post COVID-19 conditions			
			Chronic fatigue syndrome	Manipulations in respiratory system	Manipulations in cardiovascular system	Mental symptoms
T2D	24	612	61	32	2054	1223
CVD	1424	3313	1662	1507	2752	4392
Cancer	754	2160	922	821	1650	3228
Non-comorbidity		398	6	1	198	927

T2D: Type 2 Diabetes, CVD: Cardiovascular diseases.

Chronic diseases, such as cardiovascular diseases (CVDs), diabetes, and cancers were proven to aggravate the severity of COVID-19 patients [32]. Because of the huge number of drugs administered, we investigated the interaction risks between the COVID-19 drugs and the drugs used in the management of these three popular comorbidities (Table S7).

When chronic disease patients are infected with SARS-CoV-2, they may face a significantly higher risk of drug-drug interaction. For example, for a diabetic patient suffering from COVID-19, 612 potential DDI drug pairs were detected due to polypharmacy while they only have to suffer from 24 DDIs without COVID-19. Regarding cardiovascular disease and cancer, due to a larger number of drugs that may be used, there are many more drug combinations that are discovered as potential DDIs. Cancer patients are exposed to a total of 754 and 2160 potential drug interactions with and without COVID-19, relatively. Similarly, for CVD patients, the numbers are 1424 and 3313 pairs, relatively **(**Table 1**)**. Detrimental consequences derived from drug-drug interaction could be one of the important reasons resulting in severe conditions and high mortality rates in comorbid patients**.**

### 5.2 DDIs relating to the post-COVID-19 medications

After recovering from acute COVID-19 symptoms, patients with comorbidities continuously confront a high risk of drug-drug interaction regardless of the conditions patients suffer from (Table 1). For example, CVD patients who deal with long COVID-19 mental symptoms, such as generalized anxiety disorder, depression disorder, or post-traumatic stress disorder could be exposed to 4392 DDIs, which is about three-time higher than patients suffering from CVD only. When T2D patients deal with post-COVID-19 cardiovascular symptoms, there are 2054 interactions probably occurring in their prescription, which is a hundred times more than non-COVID-19 patients.

These findings could show that the high risk of DDIs not only exists at the acute infection of SARS-CoV-2 phase, but also in later phases as well. Some of these interactions could result in detrimental consequences, such as efficacy deficiency or ADR, therefore, clinicians should consider these perils before prescribing for post-COVID-19 patients.

## 6 Discussion

Although the awareness of PGx application in clinical settings for the precision therapy of COVID-19 has been raised by many experts [12,16,17], the publication of population PGx data relating to COVID-19 drugs is modest to date. Estimating the number of PharmGKB variants carried by Vietnameses could provide a landscape of risk related to COVID-19 drugs administered by Vietnamese people. Based on the number of variants recommended at the level 1 and 2 of the PharmGKB, we found a number of COVID-19 drugs which might be greatly affected by Vietnamese genetic profiles such as warfarin, the new oral anticoagulants, tocilizumab and ritonavir. Notably, these drugs are well-known for their toxicity which could result in severe adverse reactions. In addition to the actionable PharmGKB variants, in the current study, we also detected novel variants with significant frequency in the Vietnamese population which might have deleterious impacts on the therapeutic response of COVID-19 drugs. For example, the *CYP2A6* variants which influence the metabolism of two corticoids including methylprednisolone and dexamethasone, the *ABCC4* variant affecting the therapeutic response of remdesivir, or the *SLC15A1*, *SLC15A2* variants which could disrupt the transportation of many beta-lactam antibiotic such as ampicillin, cefepime, cefotaxime, and ceftriaxone.

There are a considerable difference in our COVID-19 drug list along with their relevant variants compared with the study of Sahana et al. [17] because of the dynamic change of COVID-19 medications from 2020 until 2022. Moreover, the difference indicates a distinction in the impacts of genetic polymorphisms on drug responses among various populations. In fact, the comparisons with genetic data of various populations indicated the remarkably high frequencies in the Vietnamese population of some essential actionable variants relating to the COVID-19 drug, including the *VKORC1* variants which request adjusted dosing of the VKAs, the *CYP2C19* no-function alleles which lead to impaired excretion of voriconazole, or the HLA alleles associated with severe cutaneous adverse reactions when using trimethoprim/sulfamethoxazole.

One of the novelties of the current study is the PGx revelation of the post-COVID-19 drugs which showed a much more complicated PGx landscape with 881 clinical annotations of all levels from PharmGKB associated with 83 post-COVID-19 therapies. The results showed several drugs which should be used with high caution in Vietnamese patients due to the high number of variants recommended at the level 1 and 2 of the PharmGKB. There is a wide range of them, from agents affecting the nervous system with high toxicity and narrow therapeutic windows such as those for the treatment of depressive and anxiety disorders to the OTC drugs such as acetaminophen and aspirin. We also detected novel variants with high frequency in the Vietnamese population which significantly modulate the therapeutics response of post-COVID-19 drugs. For example, a variant of the *PPARG* gene could affect the structure of such receptor and thereby the toxicity of amiodarone or several variants of the *UGT1* family which plays an important role in the phase II metabolism of angiotensin receptor blockers.

Another important contribution of the current study is the revealing of the DDI risks in patients with COVID-19 and long COVID-19, especially those with comorbidities. Due to the significantly high number of potential DDIs in polypharmacy which could worsen the condition of patients, it presents an urgent need to promote systems of pharmacovigilance to avoid the occurrence of DDIs and their detrimental consequences. A recent study based on FDA Adverse Event Reporting System detected 424 DDI signals related to 176 drug pairs on 13 COVID-19 drugs and 60 comorbid drugs [62]. In the current study, given the increased risk posed by co-administration in severe COVID-19 patients with chronic disorders, we found that patients with each of three underlying morbidities are at an increased risk of DDIs when dealing with COVID-19. This result could explain for observation of Ramírez et al. that COVID-19 patients are facing a 4.75-fold higher incidence of adverse drug reactions (ADRs) compared to non-COVID-19 patients. Among three conditions, diabetic patients have the highest interaction risk related to shared pharmacogenes when added COVID-19 drugs in the regimen. While COVID-19 drugs pose a lower interaction risk in cardiovascular and cancer patients. The use of computational and network biology methods for the analysis of potential DDIs have been developed recently and provide a powerful tool for the analyses of a huge number of drug pairs in such a complicated case of polypharmacy in COVID-19 or post-COVID-19 patients with existing chronic diseases [63].

Our study was carried out by using a large sample size of 1008 whole genome sequences, partially filling the gaps of genetic information in Vietnamese people in particular and Asian populations in general. Thereby, this study presented valuable insights related to pharmacogenomic essences of several common drug groups not only used in COVID-19 treatment, but also in multiple other disorders. We constructed a comprehensive landscape including SNPs, indels, star alleles and HLA alleles, along with a prediction model for DDIs in complicated diseases like COVID-19 using different bioinformatic tools, that could be a reference framework for assessing pharmacogenomic data in other pharmacological groups. Also, our current results created some very first signals of the influences of genetic variants on responses to many drugs for following studies to get insights. Nonetheless, as a population genetic study, these results were generated by using data from healthy individuals, which could pose a number of differences with patients. Therefore, it is required further association studies in patients to validate these annotations prior to implementing in clinical practice.

## 7 Conclusion

Our study has revealed the potential genetic-related risk of adverse response to multiple drug groups in Vietnamese population, such as tocilizumab, ritonavir, dexamethasone in COVID-19 treatment and SSRIs, aspirin and acetaminophen in post-COVID-19 treatment. An increased risk of DDIs was also observed in COVID-19 patients with three common comorbidities, type 2 diabetes, cardiovascular disease, and cancers. The results of the current study could help to orientate the COVID-19 research toward improving therapeutic outcomes by maximizing the efficacy and safety of the treatment regimens.

## Funding

This work was supported by the Vingroup Big Data Institute.

## Ethics approval statement

In the 1KVG study, subjectsprovided informed consent and the study was approved by the Vinmec International Hospital Institutional Review Board with number 543/2019/QƉ-VMEC. out in accordance with the relevant guidelines and regulations (e.g. Helsinki Declaration).

## Data availability statement

The 1KGP phase 3 (https://www.internationalgenome.org/) are publicly available on the internet. The VN1K WGS and genotyping datasets are available under agreement at MASH data portal (https://genome.vinbigdata.org/). All the allele frequencies of investigated variants are available in the Supplementary file.

## CRediT authorship contribution statement

**Thien Khac Nguyen:** Data curation, Formal analysis, Investigation, Writing – original draft, Writing – review & editing. **Giang Minh Vu:** Data curation, Formal analysis. **Vinh Chi Duong:** Data curation, Formal analysis. **Thang Luong Pham:** Formal analysis. **Nguyen Thanh Nguyen:** Formal analysis. **Trang Thi Ha Tran:** Resources. **Mai Hoang Tran:** Resources. **Duong Thuy Nguyen:** Formal analysis. **Nam S. Vo:** Conceptualization, Resources. **Huong Thanh Phung:** Conceptualization, Data curation, Formal analysis, Writing – original draft, Writing – review & editing. **Tham Hong Hoang:** Conceptualization, Data curation, Formal analysis, Investigation, Supervision, Writing – original draft, Writing – review & editing.

## Declaration of competing interest

The authors declare that they have no known competing financial interests or personal relationships that could have appeared to influence the work reported in this paper.

## Abbreviations

1KVG: 1000 Vietnamese Genomes Project
1KGP3: 1000 Genome Project Phase 3
ADR: adverse drug reaction
COVID-19: Coronavirus disease 2019
CTET: carriers, transporters, enzymes, and targets
CVD: Cardiovascular disease
CYP: cytochrome P450
DDI: drug-drug interaction
gnomAD: Genome Aggregation Database
NICE: the U.K National Institute for Health and Care Excellence
NOAC: new oral anticoagulants
NSAID: Non-steroidal anti-inflammatory drugs
PGx: Pharmacogenomics
PharmGKB: Pharmacogenomics Knowledge Base
OTC: Over-the-counter
SARS-CoV-2: Severe acute respiratory syndrome coronavirus 2
SJS: Stevens-Johnsons syndrome
SNP: single nucleotide polymorphism
VCF: Variant Calling Format
WHO: World Health Organization
TEN: Toxic Epidermal Necrolysis
